This article has been retracted.

# MicroRNA-21 promotes TGF-β1-induced epithelial-mesenchymal transition in gastric cancer through up-regulating PTEN expression

**DOI:** 10.18632/oncotarget.11888

**Published:** 2016-09-07

**Authors:** Chang Li, Lei Song, Zhuo Zhang, Xiao-Xue Bai, Ming-Fu Cui, Lian-Jun Ma

**Affiliations:** ^1^ Department of Gastrointestinal Surgery, China-Japan Union Hospital of Jilin University, Changchun, 130000, Jilin, P.R. China; ^2^ Department of Respiratory Medicine, The First Hospital of Jilin University, Changchun, 130000, Jilin, P.R. China; ^3^ Department of Orthopaedics, China-Japan Union Hospital of Jilin University, Changchun, 130000, Jilin, P.R. China; ^4^ Department of Cadre Ward, The First Hospital of Jilin University, Changchun, 130000, Jilin, P.R. China; ^5^ Department of Endoscopics, China-Japan Union Hospital of Jilin University, Changchun, 130000, Jilin, P.R. China

**Keywords:** gastric cancer, epithelial-mesenchymal transition, MicroRNA-21, PTEN, TGF-β1

## Abstract

This study aimed to explore the effects of miR-21 and PTEN/Akt signaling pathway on TGF-β1-induced epithelial-mesenchymal transition (EMT) in gastric cancer (GC). GC tissues and adjacent tissues were collected from 83 patients. The qRT-PCR assay was performed to detect miR-21 expression. The expressions of PTEN, Akt and p-Akt were detected by immunohistochemistry. After 48 h of treatment with TGF-β1 (10 ng/mL), the SGC-7901 and KATO-III cells were divided into the blank, negative control (NC), miR-21 inhibitors, PTEN-siRNA and miR-21 inhibitors + PTEN-siRNA groups. EMT related factors and PTEN expressions were detected by qRT-PCR assay and Western blotting. The scratch test was conducted to observe cell migration. Xenograft tumor model in nude mice was used to evaluate the effects of miR-21 on EMT of GC cells *in vivo*. In GC tissues, the expressions of miR-21, Akt and p-Akt were up-regulated, while PTEN expression was down-regulated. Gene and protein expressions of E-cadherin and PTEN in the miR-21 inhibitors group were higher than the blank, NC, PTEN-siRNA and miR-21 inhibitors + PTEN-siRNA groups, while the expressions of N-cadherin, β-catenin, Vimentin and Slug in the miR-21 inhibitors group were lower than other groups. MiR-21 inhibitors significantly inhibit cell migration and invasion in GC cell lines. *In vivo* xenograft experiment revealed that miR-21 inhibitor inhibits the growth of transplanted tumor through up-regulating E-cadherin and PTEN expressions and down-regulating the expressions of N-cadherin, β-catenin, Vimentin and Slug. These results suggest that miR-21 could promote TGF-β1-induced EMT in GC cells through up-regulating PTEN expression.

## INTRODUCTION

Gastric cancer (GC) is one of the most common malignant tumors of digestive system. It is estimated that 0.989 million new GC cases occured in 2008 and 0.738 million GC deaths occur every year worldwide [1–2]. With study on the molecular biological mechanism of GC appearing, developing and transiting, targeted drug therapy for GC attracted more concern in clinical trials [3]. The pathogenic factors of GC include environmental factors, diet, infections and host genes, among which the abnormalities in gene expression, especially the abnormal expression of the encoded protein of oncogenes or tumor-suppressor genes, play an important role in the pathogenesis of GC [4, 5]. Epithelial-mesenchymal transition (EMT) in GC is the key factor for GC cell metastasis and also is the primary cause of GC death. Hence study on gene regulation mechanism of EMT in GC has great significance [6].

Molecular target technology has been widely used in the study of GC and microRNA (miR) is one of the most common molecular targets which have been applied to the diagnosis, treatment and prognosis of GC [7]. It is presumed that about one third of the human genes are regulated by miRs [8]. MiR-21 is highly expressed in multiple cancers, such as epithelial cell cancer, connective tissue cancer, hematopoietic cell cancer, reproductive cell cancer and nerve cell cancer [9]. Previous studies have demonstrated that the target genes of miR-21 including phosphatase and tensin homolog detected on chromosome 10 (PTEN), *Bcl-2*, *TPM1* and *PDCD4* which are cancer suppressed genes [10–13]. Previous studies have shown that miR-21 regulates PTEN by interacting with its target gene *3′-UTR* and participates in the process of cancer occurrence and development [14–15]. In current study, we aim to investigate the role of miR-21 and its target gene PTEN in TGF-β1-induced EMT in GC and to search for new molecular therapy targets for GC.

## RESULTS

### Expressions of miR-21, PTEN, Akt and p-Akt in gastric cancer and adjacent normal tissues

The expressions of miR-21 and PTEN in GC tissue were higher than those in adjacent normal tissue (4.25 ± 1.09 vs. 0.86 ± 0.11, *P* < 0.05) (Figure 1A). The Akt and p-Akt expressions in GC tissue were also significantly higher than those in adjacent normal tissue (all *P* < 0.05) (Figure 1B). Immunohistochemistry staining showed that PTEN was mainly found in cytoplasm and cytomembrane, while Akt and p-Akt mainly in the nucleus (Figure 2). As shown in Table 3, the expressions of miR-21 and PTEN showed significant associations with lymph node metastasis, differentiation grade and TNM stage of GC patients (all *P* < 0.05). However, both miR-21 and PTEN expressions exhibited no associations with age and gender of GC patients (both *P* > 0.05). The correlation analysis demonstrated that there was a negative correlation between miR-21 and PTEN in GC (*r* = −0.865, *P* < 0.01), while positive correlations were found between miR-21 and Akt/ p-Akt in GC (Akt: *r* = 0.747, *P* < 0.001; pAkt: *r* = 0.804, *P* < 0.01).

**Figure 1:** The expressions of miR-21, PTEN, Akt and p-Akt in GC tissue and adjacent normal tissue (**A**) The expression of miR-21 in GC tissue and adjacent normal tissue detected by qRT-PCR assay. (**B**) The expressions of PTEN, Akt and p-Akt in GC tissue and adjacent normal tissue detected by immunohistochemistry). Note: GC, gastric cancer; qRT-PCR, real-time polymerase chain reaction; *comparison with adjacent normal tissue, *P* < 0.05.

**Figure 2:** Immunohistochemistry images of the expressions of PTEN, Akt and p-Akt in GC tissue and adjacent normal tissue (× 400) (**A**, **B**, **C**) The expressions of PTEN, Akt and p-Akt in GC tissue. (**D**, **E**, **F**) The expressions of PTEN, Akt and p-Akt in adjacent normal tissue). Note: GC, gastric cancer.

### Targeting regulatory relation between miR-21 and PTEN

Target Scan was used to ensure the target site of PTEN combining with miR-21 and the 3′-UTR sequence of PTEN mRNA combining with miR-21, which were shown in Figure 3A. In PTEN-3′-UTR-WT transfection group, after transfected with miR-21 inhibitors, the relative activity of luciferase significantly increased compared with the NC groups (PTEN-3′-UTR-WT+NC group and PTEN-3′-UTR-MT group) (all *P* < 0.05) (Figure 3B). After PTEN-3′-UTR-MT group was transfected with miR-21 inhibitors, the comparison of relative activity of luciferase between PTEN-3′-UTR-MT and PTEN-3′-UTR-MT+NC groups showed no statistical difference (*P* > 0.05) (Figure 3B). These results demonstrated that PTEN was the target gene of miR-21.

**Figure 3:** PTEN is the target gene of miR-21 (**A**) miR-21 combined with PTEN 3′UTR; (**B**) the activity assay of dual luciferase reporter gene, activity assay of luciferase correlated with miR-21 inhibitors and PTEN 3′UTR WT/MT in gastric cancer cells, miR-21inhibited the luciferase activity of WT plasmid but it had no influence on that of MT plasmid). Note: *compared with the control group, *P* < 0.05).

### TGF-β1 induced EMT in GC and altered the expressions of miR-21 and PTEN

After TGF-β1 treatment for 48 h, immunofluorescence staining showed that E-cadherin expression was significantly reduced (Figure 4). However, high expression of E-cadherin was observed in SGC-7901 and KATO-III cells without TGF-β1 treatment. After TGF-β1 treatment, the miR-21 expression was remarkably higher than that in the BSA control group, while PTEN mRNA expression was significantly reduced in both SGC-7901 and KATO-III cells (all *P* < 0.05) (Figures 5A and 6A). Compared with the BSA control group, the mRNA expressions of N-cadherin, β-catenin, Vimentin and Slug up-regulated and E-cadherin mRNA expression down-regulated after TGF-β1 treatment in both SGC-7901 and KATO-III cells (all *P* < 0.05) (Figures 5B and 6B). Western blotting also showed that the E-cadherin expression down-regulated but the expressions of N-cadherin, β-catenin, Vimentin and Slug up-regulated after TGF-β1 treatment in both SGC-7901 and KATO-III cells (all *P* < 0.05) (Figures 5C, 5D and 6C, 6D).

**Figure 4:** Immunofluorescence staining of E-cadherin expression in SGC-7901 and KATO-III cells after TGF-β1 treatment for 48 h (×200) (**A**) E-cadherin expression in SGC-7901 cells in the BSA control group; (**B**) E-cadherin expression in SGC-7901 cells with TGF-β1 treatment; (**C**) E-cadherin expression in KATO-III cells in the BSA control group; (**D**) E-cadherin expression in KATO-III cells with TGF-β1 treatment). Note: TGF-β1, transforming growth factor β1; GC, gastric cancer; BSA, bovine serum albumin.

**Figure 5:** The influences of TGF-β1 treatment on the expressions of miR-21, PTEN and EMT related factors in SGC-7901 cells (**A**) The expressions of miR-21 and PTEN detected by qRT-PCR assay; (**B**) The mRNA expressions of EMT related factors detected by qRT-PCR assay; (**C**–**D**) The protein expressions of of EMT related factors detected by Western blotting). Note: TGF-β1, transforming growth factor β1; BSA, bovine serum albumin; EMT, epithelial-mesenchymal transition; *comparison with BSA control group, *P* < 0.05.

**Figure 6:** The influences of TGF-β1 treatment on the expressions of miR-21, PTEN and EMT related factors in KATO-III cells (**A**) The expressions of miR-21 and PTEN detected by qRT-PCR assay; (**B**) the mRNA expressions of EMT related factors detected by qRT-PCR assay; (**C**–**D**) The protein expressions of of EMT related factors detected by Western blotting). Note: TGF-β1, transforming growth factor β1; BSA, bovine serum albumin; EMT, epithelial-mesenchymal transition; *,comparison with the BSA control group, *P* < 0.05.

### miR-21 inhibited TGF-β1-induced EMT in GC

After transfection of miR-21 inhibitors, the miR-21 expression of SGC-7901 and KATO-III cells in the miR-21 inhibitors group and miR-21 inhibitors + PTEN-siRNA group decreased (all *P* < 0.05), while no significant change was found in other three groups (all *P* > 0.05) (Figure 7). After TGF-β1 treatment, both SGC-7901 and KATO-III cells in the miR-21 inhibitors group had cobblestone-like morphology and were conjunct with each other closely (Figure 8); the cells in the PTEN-siRNA group and miR-21 inhibitors + PTEN-siRNA group had long ectomesenchymal spindle shape, were dispersed and had migration synapse which were more obvious compared with the blank group and the NC group. The immunofluorescence staining showed that the E-cadherin expression in the miR-21 inhibitors group was apparently higher than that in the blank group and the NC group; the E-cadherin expressions in PTEN-siRNA group and miR-21 inhibitors + PTEN-siRNA group lowered significantly.

**Figure 7:** The miR-21 expression in SGC-7901 and KATO-III cells after cell transfection Note: *comparison with the blank group, negative normal group or PTEN-siRNA group, *P* < 0.05).

**Figure 8:** The morphological changes of SGC-7901 and KATO-III cells after TGF-β1 treatment and the effects of TGF-β1 on E-cadherin expression (×200) (**A**–**E**) The E-cadherin expression in SGC-7901 cells in the blank group, negative control group, miR-21 inhibitors group, PTEN-siRNA group and miR-21 inhibitors + PTEN-siRNA group; (**F**–**J**) the E-cadherin expression in KATO-III cell in the blank group, negative control group, miR-21 inhibitors group, PTEN-siRNA group and miR-21 inhibitors + PTEN-siRNA group).

The results of qRT-PCR assay and Western blotting showed that gene and protein expressions of E-cadherin in SGC-7901 cells in the miR-21 inhibitors group was higher than those in the blank and NC groups, while E-cadherin expression in the PTEN-siRNA and miR-21 inhibitors + PTEN-siRNA groups reduced significantly compared with the blank and NC groups (all *P* < 0.05) (Figure 9A–9C). However, compared with the blank and NC groups, gene and protein expressions of N-cadherin, β-catenin, Vimentin and Slug in SGC-7901 cells in the miR-21 inhibitors group down-regulated, while up-regulations of N-cadherin, β-catenin, Vimentin and Slug expressions were observed in the in the PTEN-siRNA and miR-21 inhibitors + PTEN-siRNA groups (all *P* < 0.05). The gene and protein expressions of EMT related factors in KATO-III cells in each group were consistent with those in SGC-7901 cells (Figure 9D–9F).

**Figure 9:** The mRNA and protein expressions level of EMT related factors in SGC-7901 and KATO-III cells after induced by TGF-β1 for 48 h (BL, blank group; NC, negative control group; IN, miR-21 inhibitors group (**A**) The analysis histogram of mRNA expression of EMT related factors in SGC-7901 cells; (**B**) The expression of EMT related factors in SGC-7901 cells tested by Western blot; (**C**) The analysis histogram of EMT related factors in SGC-7901 cells; (**D**) The analysis histogram of mRNA expression of EMT related factors in KATO-III cells; (**E**) the expression of EMT related factors in KATO-III cells tested by Western blot; (**F**) the analysis histogram of EMT related factors in KATO-III cells; TGF-β1, transforming growth factor β1; EMT, epithelial-mesenchymal transition; *comparison with the blank group and NC group, *P* < 0.05; #,comparison with IN group, *P* < 0.05).

### Alterations of PTEN/Akt signal pathway after TGF-β1 treatment and cell transfection

After cell transfection and TGF-β1 treatment for 48 h in SGC-7901 and KATO-III cells, gene and protein expressions of PTEN in the miR-21 inhibitors group were significantly higher than that in the blank group and the NC group (both *P* < 0.05), while PTEN expressions in the PTEN-siRNA and miR-21 inhibitors + PTEN-siRNA groups were lower than that in the blank and the NC groups (all *P* < 0.05) (Figure 10). No significant differences in Akt gene and protein expressions were observed among the five groups (all *P* > 0.05). The gene and protein of p-Akt in the miR-21 inhibitors group was significantly lower than those in the blank and the NC group (all *P* < 0.05), while p-Akt expressions in the PTEN-siRNA and the miR-21 inhibitors + PTEN-siRNA groups were up-regulated significantly compared with the blank group and the NC group (all *P* < 0.05).

**Figure 10:** The gene and protein expressions of PTEN, Akt and p-Akt in SGC-7901 and KATO-III cells after cell transfection and TGF-β1 treatment for 48 h (**A**–**C**) PTEN, Akt and p-Akt expressions in SGC-7901 cells; (**D**–**F**) PTEN, Akt and p-Akt expressions in KATO-III cells). Note: *comparison with the blank group and NC group, *P* < 0.05; #comparison with the IN group, *P* < 0.05.

### Cell migration after TGF-β1 treatment

After cell transfection and TGF-β1 treatment for 48 h in SGC-7901 and KATO-III cells, compared with the blank group and the NC group, cell migration and invasion in the miR-21 inhibitors group decreased significantly (all *P* < 0.05), while in the PTEN-siRNA and miR-21 inhibitors + PTEN-siRNA group increased evidently (all *P* < 0.05). There was no obvious difference in cell migration and invasion between the blank group and the NC group (*P* > 0.05) (Figure 11). The scratch test showed that miR-21 inhibitors significantly inhibit cell migration and invasion in GC cell lines

**Figure 11:** A scratch test for evaluating cell migration and invasion in SGC-7901 and KATO-III cells after cell transfection and TGF-β1 treatment for 48 h (**A**) scratch test of SGC-7901 cells in each group; (**B**) scratch test of KATO-III cells in each group).

### Tumorigenesis and growth of xenograft in nude mice

Nude mice in the blank and NC groups inoculated with SGC-7901 cells presented tumorigenesis after about 10 days, while mice in the miR-21 inhibitors group showed tumorigenesis 12 days after inoculation or even later, with tumors growing slowly. After tumorigenesis, tumors in the blank group and the NC group grew rapidly and tumor volume was obviously larger than that in the miR-21 inhibitors group (*P* < 0.05) (Figure 12A). The results showed that tumor weight of mice in the miR-21 inhibitors group was significantly lower than that in the blank group and the NC group (all *P* < 0.05) (Figure 12B).

**Figure 12:** Xenograft tumor model in nude mice by inoculation with SGC-790 cell lines (**A**) The growth curve of xenograft in each group; (**B**) tumor weight of xenograft in each group).

### Effects of miR-21 on the expressions of EMT related factors and PTEN of xenograft in nude mice

Immunofluorescence results demonstrated that the expressions of E-cadherin and PTEN proteins in the miR-21 inhibitors group increased significantly, while the expressions of N-cadherin, β-catenin, Vimentin and Slug decreased remarkably compared with the blank group and the NC group (all *P* < 0.05). These results suggested that miR-21 inhibitors could inhibit the growth and proliferation of xenograft through up-regulating E-cadherin and PTEN expressions and down-regulating N-cadherin, β-catenin, Vimentin, and Slug expressions (Figure 13).

**Figure 13:** The expressions of EMT related factors(E-cadherin, N-cadherin, β-catenin, Vimentin, Slug) and target gene PTEN of xenograft in nude mice

## DISCUSSION

In the present study, our results demonstrated that the expressions of miR-21, Akt and p-Akt were significantly higher in the 83 GC tissues than those in adjacent normal tissues, but the expression of PTEN was significantly lower than that in adjacent normal tissue, which indicated that the expressions of miR-21, Akt, p-Akt and PTEN were related to GC. The further analysis of GC patients with different lymph node metastasis, tumor differentiation and TNM stage showed that PTEN expression was lower in GC patients with no or low differentiation, had lymph node metastasis and at TNM III/IV stage. The study has found that the PTEN expression level in normal gastric mucosa was higher than that in GC tissues and the PTEN expression level dropped with the decrease of differentiation degree [16]. It was reported that the positive rate of PTEN expression decreased with the deeper infiltrating degree, the lower differentiation degree and lymph node metastasis, which indicated that PTEN was possibly participated in the occurrence and development of GC [16]. The regulation of PTEN expression was not clear and it was considered that heterozygosity loss, mutations, promoter methylation and microRNA regulation of PTEN were the reasons for PTEN's participation in GC [17]. Furthermore, the correlation analysis demonstrated a negative correlation between miR-21 and PTEN expression level, while a positive correlation between miR-21 and Akt expression level, and between miR-21 and p-Akt expression level. To further explore the mechanisms of PTEN involved in GC, the study used miR-21 targeted molecular technique and identified PTEN as the target gene of miR-21 through online prediction and transfection with miR-21 inhibitors. Meng et al. showed that if miR-21 was inhibited, its target gene PTEN expression would up-regulate and the growth, migration and invasion of cancer cells would decrease [14]. After miR-21 in keratinocytes was cleaned away, PTEN would rise [18]. All these indicated that miR-21 could regulate the occurrence of GC though down-regulating PTEN. After TGF-β1 treatment, the miR-21expression was remarkably higher than that in the control group while PTEN mRNA expression was significantly lowered

EMT improved the abilities of cancer cells' migration, invasion, anti-apoptosis and extracellular matrix degradation [18]. In our study, we built a model of EMT in GC to explore the pathogenesis of GC. TGF-β1 was the most effective inductor for EMT and was confirmed as the main cytokines of promoting fibrosis [19]. The study results showed that TGF-β1 induced the EMT in GC cell, and cell morphology changed from polygon to long ectomesenchymal spindle shape and cells were dispersed even with migration synapse. Immunofluorescence showed that the expression of E-cadherin lowered and the expression of N-cadherin, β-catenin, Vimentin and Slug rose.

In the model of TGF-β1-mediated EMT in GC, the study found that miR-21 promoted phosphorylation of Akt through dropping PTEN which promote the EMT in GC induced by TGF-β1. The study of Wei also found that PTEN negatively regulated Akt and lowered Akt phosphorylation level [20]. Meadow' study found that Akt promote the EMT [21]. Its mechanism may be that PTEN had phosphatase activity and its role was to make the second messenger PIP3 dephosphorylated phosphatidylinositol, then generated PIP2 and lowered phosphorylation levels of Akt [22]. Akt makes glycogen synthase kinase 3β (GSK3β) lose the kinase activity which promotes the activity of transcription factor Snail and Slug, further inhibited E- cadherin expression and then caused EMT [23]. The mechanism of GSK3β inhibition of Snail and Slug was phosphorylation which makes Snail and Slug transferred from nucleus to cytoplasm and thereby was degraded by ubiquitinated [24]. Moreover, Akt pathway promoted EMT by enhancing the transcriptional activity of hypoxia-inducible factor-1α (HIF-1α). On one hand, HIF-1α could accelerate tumor metastasis by affecting the expression of tumor cell adhesion molecules, such as E-cadherin and β-catenin [25]. On the other hand, HIF-1α could cause the expression of matrix metalloproteinases (MMPs) and thus promoted tumor metastasis [26].

Moreover, we conducted a xenograft tumor experiment in nude mice, with cell migration detected by scratch test, tumorigenesis and growth of xenograft observed, and effect of miR-21 on EMT related transcription factors in subcutaneous xenograft in nude mice analyzed. The results demonstrated that compared with the blank group and the NC group, wound healing rate in the miR-21 inhibitors group decreased significantly, while in the PTEN-siRNA group and the miR-21 inhibitors + PTEN-siRNA group increased evidently. In addition, tumor weight in the miR-21 inhibitors group (both GC SGC-7901 and KATO-III cell lines) was significantly lower than that in the blank group and the NC group, which indicated that miR-21 inhibitors could inhibit the growth of subcutaneous xeongraft in GC SGC-7901 and KATO-III cell lines. Moreover, the expressions of E-cadherin and PTEN proteins in the miR-21 inhibitors group increased significantly while the expressions of N-cadherin, β-catenin, Vimentin and Slug proteins decreased remarkably compared with the blank group and the NC group, suggesting that miR-21 inhibitors might inhibit the growth and proliferation of xenograft through up-regulating E-cadherin and PTEN protein expressions and down-regulating N-cadherin, β-catenin, Vimentin, and Slug protein expressions.

In a word, this study found that TGF-β1 can induce EMT in GC cells, and up-regulate miR-21 while down-regulate PTEN; and miR-21 expression inhibition can promote the phosophorylation of AKt and inhibit EMT through up-regulating target gene PTEN, which was further verified by an *in vivo* experiment using a xenograft model in nude mice. Therefore, we may conclude that miR-21 could promote TGF-β1-induced EMT in GC cells through up-regulating PTEN expression. The study laid theoretical foundation for studying the molecular mechanism and new therapeutic targets of GC.

## MATERIALS AND METHODS

### Ethical statement

This study was approved by the Ethics Committee of China-Japan Union Hospital of Jilin University and all experimental methods were performed in accordance with the Declaration of Helsinki. All study participants provided written informed consent before the experiments.

### Subjects

Specimens were collected from 83 patients with GC who received surgical treatment in the China-Japan Union Hospital of Jilin University from June 2014 to January 2015. All specimens were confirmed by pathological diagnosis. Among the 83 patients (53 male and 30 female; mean age, 53.6 ± 12.5 years), 47 cases were less than 60 years old and 36 cases were equal to or older than 60 years old; 49 cases were middle-differentiated or well-differentiated, and 34 cases were low-differentiated or non-differentiated. According to tumor node metastasis (TNM) stage recommended by the American Joint Committee on Cancer (AJCC) in 2010 [27]: 39 cases were at I/II stages, and 44 cases were at III/IV stages. There were 38 cases without lymph node metastasis, and 45 cases had lymph node metastasis. All patients did not receive chemotherapy or radiotherapy before the experiment. The GC tissue and adjacent normal tissue (5 cm away from cancer tissue) were collected and stored at −70°C after processing by liquid nitrogen. Half of the specimens were used for measurement of miR-21 expression and the other half were fixed by 10% formalin and embedded in paraffin for immunohistochemistry.

### qRT-PCR assay

The quantitative real-time polymerase chain reaction (qTR-PCR) assay was performed to detect the expression of miR-21 in tissues. The tissue specimens were sliced and pulverized by the liquid nitrogen grounding method. Total RNA was extracted from tissue specimens by Trizol one-step method (Invitrogen, USA) and dissolved by ultrapure water which was processed by diethylpyrocarbonate (DEPC). The quality of total RNA was identified by measuring absorbance of 260 nm and 280 nm with ND-1000 UV/VIS spectrophotometer (NanoDrop Technologies, USA). According to kit instructions (USA Fermentas Corporation), the RNA was extracted from tissues and cells were reversely transcribed. The reaction conditions were: 70°C for 10 min, ice bath for 2 min, 42°C for 60 min, 70°C for 10 min, and then cDNA was temporarily placed at −80°C. The primer sequences were shown in Table 1. The reaction conditions were: pre-denaturation at 95°C for 30 s, denaturation at 95°C for 10 s, annealing at 60°C for 20 s and extension at 70°C for 10 s, which were cycled for 40 times. The test was performed using qRT-PCR (Bio-Rad iQ5; Bio-Rad Laboratories, Hercules, Calif., USA). The internal reference of miR-21 was U6 and that of other target genes was β-actin. The relative quantification method was used for calculation and 2^−ΔΔCt^ was used to represent the relative multiple expressions of target genes. All experiments were repeated for 3 times.

**Table 1:** miR-21 and PTEN expressions in gastric cancer patients

	*n*	miR-21 expression	*P* value	PTEN expression	*P* value
Age					
≥ 60	36	2.84 ± 0.89	0.96	38.9%	0.78
< 60	47	2.83 ± 1.23		55.3%	
Gender					
Male	53	2.79 ± 1.09	0.97	60.0%	0.51
Female	30	2.80 ± 1.11		41.5%	
Lymph node metastasis					
Yes	45	4.91 ± 0.85	< 0.001	17.8%	< 0.001
No	38	3.47 ± 0.79		84.2%	
Differentiation grade					
Well-differentiated	49	3.59 ± 0.72	< 0.001	71.4%	0.001
Poorly differentiated	34	5.20 ± 0.78		14.7%	
TNM stages					
I/II	39	4.94 ± 0.83	< 0.001	84.6%	< 0.001
III/IV	44	3.47 ± 0.78		15.9%	

Note: TNM, tumor node metastasis.

### Immunohistochemistry

The protein expressions of PTEN, Akt and p-AKT was tested by PV-9000 two-step method. Every tissue microarray wax block was cut into slices (4 μm) and the slices were dewaxed to gradient alcohol hydration and repaired by antigen microwave. Endogenous peroxidase was blocked by 3% hydrogen peroxide, and then primary antibodies [mouse anti-human PTEN, mouse anti-human Akt, and mouse anti-human p-AKT; all 1:500 (Framingham, Massachusetts, USA)] were added and stored at 4°C overnight. The slices were incubated at room temperature for 20 min after added with polymerase auxiliary agent, and then 30 min after added with horseradish peroxidase labeled goat anti-mouse second antibody (Abcam, UK), and dyed bydiaminobenzidine (DBA) (Sigma, USA). The slices were re-dyed by hematoxylin and then sealed. PBS was selected as a negative control and adjacent normal tissue as a positive control. The positive expression of PTEN protein was presented in yellow brown in cytoplasm and the positive expression of Akt protein was yellow brown or brown in nucleus. Each slice was observed by four high power fields (× 400) with 200 cells counted in each field. The immunohistochemistry score was assessed according to percentage of positive cells: positive tumor cells/tumor cells > 10% was marked positive (+); positive tumor cells ≤ 10% was marked negative (−). As for Akt, if the nucleus had brown granules, it was positive. Five high power fields were randomly selected and percentage of positive cells was used as tagged value of Akt. The percentage of positive cells > 10% was positive (+) and the percentage of positive cells ≤ 10% was negative (−) [28]. Immunohistochemistry result was scored using double-blind method by two independent investigators.

### Cell culture

SGC-7901 cells (purchased from Shanghai Cell Bank of Chinese Academy of Sciences) and KATO-III cells (purchased from ATCC Co., Ltd., USA) were cultured in Thermo Scientific 8000 carbon dioxide incubator (Thermo Scientific) using Roswell park memorial institute (RPMI) 1640 culture medium (Gibco Company, Carlsbad, USA) containing 10% bovine serum albumin (BSA) (Hyclone, USA) under 5% CO_2_ and 95% humidity at 37°C. Cultured cells had monolayer growth and rate of cells passaging the attachment reached 90%. At the time of passage, pour conventional culture medium was poured and the samples were washed with PBS (twice) and digested with 0.25% trypsin (Gibco Company, Carlsbad, USA). After cell gap increased, trypsin was removed and RPMI-1640 culture medium with 10% fetal bovine serum was used to make cells into single-cell suspension until the cells were passaged regularly.

### Luciferase reporter gene assay

According to various online analysis software of miRNA target gene, such as TargetScan, miRanda, miRbase and Pictar, the possible target gene of miRNA were predicted and gene fragments with action site were obtained. The deoxyribosenucleic acid (DNA) of GC cells was extracted according to TIANamp Genomic DNA Kit instruction (TIANGEN BiotechCo., Ltd., Beijing, China). The natural PTEN 3′UTR sequence was PTEN-3′-UTR-WT, and the mutation sequence of PTEN 3′UTR without miR-21 binding site was PTEN-3′-UTR-MT (as shown in Table 2). Luciferase reporter gene vector was established and GC cells were transfected. Luciferase reporter gene detection reagent (Promega Company, San Luis Obispo, USA) was used to test the activity of Luciferase. After transfected for 48 h, previous culture medium was removed, the samples were washed twice with PBS and added with 100 μl passive lysis buffer (PLB), followed by shakeing slightly for 15 min to get the lysis solution. The procedure was set as prereading 2 s, reading 10 s and every sample volume of LARII and Stop & Glo^®^ Reagent (TurnerBioSystems Company, UBA) was 100 μl. The prepared LARII and Stop & Glo^®^ Reagent (both 20 μl) were added into the lysis solution and then the test was performed by bioluminescent detector (Turner Biosystems Company, UBA, Model Number Modulus™).

**Table 2:** Primer sequence for quantitative real-time polymerase chain reaction (qTR-PCR) assay

Target gene	Primer sequence
miR-21	F: 5′-ACACTCCAGCTGGGTAGCTTAT-3′
	R: 5′-TGGTGTCGTGGAGTCG-3′
U6	F: 5′-CTGCTTCGGCAGCACA-3′
	R: 5′-AACGCTTCACGAATTTGCGT-3′
E-cadherin	F: 5′- CAACGACCCAACCCAAGAA-3′
	R: 5′- CCGAAGAAACAGCAAGAGCA-3′
N-cadherin	F: 5′-TTGGTTTGGGGAGGGAGA-3′
	R: 5′-CTGGGGTCAGAGGTGTATCATTT-3′
β-catenin	F: 5′-TGCCAAGTGGGTGGTATAGAGG-3′
	R: 5′-CGCTGGGTATCCTGATGT-3′
Vimentin	F: 5′-GGCTCAGATTCAGGAACAGC-3′
	R: 5′-GCTTCAACGGCAAAGTTCTC-3′
Slug	F: 5′-CAAGGACACATTAGAACTCACAC-3′
	R: 5′-CTACACAGCAGCCAGATTC-3′
PTEN	F: 5′-CCAAGCTTATGACAGCCATCATC-3′
	R: 5′-CGCGGATCCTCAGACTTTTGTAA-3′
β-actin	F: 5′-GAATCAATGCAAGTTCGGTTCC-3′
	R: 5′-TCATCTCCGCTATTAGCTCCG-3′

Note: F, forward; R, reverse.

**Table 3:** The seed sequence of miR-21 matched the 3′UTR of PTEN gene

Type	Sequence
PTEN-3′-UTR-WT	F: 5′-TTGTGGCAACAGATAAGTTTGCAGTTGGCTAAGAGAGGTT-3′
	R: 5′-CATTCCCCTAACCCGAATACATGCATTAGAATGTAGCAAA-3′
PTEN-3′-UTR-MT	F: 5′-TTGTGGCAACAGCTGAATCTGCAGTTGGCTAAGAGAGGTT-3′
	R: 5′-ATGTAGCAAAACCCTTCGGAAACCTCTCTTAGCCAACTGC-3

Note: F, forward; R, reverse.

### TGF-β1 induced cells and immunofluorescence assay

The SGC-7901 and KATO-III cells were seeded into appropriate culture plates with 5 × 10^4^/cm^2^. When grown to subconfluence, cells were washed three times with serum-free RPMI-1640 and serum starved for 24 h at 37°C. The cells were washed once again with serum-free RPMI-1640 and TGF-β1 (Sigma Company, USA) with a final concentration of 10 ng/ml was used to induce cells for 48 h and 10 ng/ml BSA (Sigma Company, USA) was used as the control. The processed cells were washed with PBS twice. Firstly, 4% paraformaldehyde (Beijing Solarbio Corporation) were added into the cells and then the cells were put at room temperature for 20 min. Secondly, 0.3% TritonX-100 (Beijing Solarbio Corporation) were added and then they were put at room temperature for 10 min. Lastly, 5% BSA 800 μl were added and then they were put at room temperature for 1 h. E-cadherin antibody (CST company, US) diluted by 5% BSA according to the proportion of 1:200 was added and then the cells were incubated at 4°C overnight. The cells were washed with PBS next day. Phycoerythrin (PE)-labeled rabbit anti-mouse secondary antibody (Abcam Company, UK) was diluted by 5% BSA (1:1000) and then cells were incubated at room temperature away from light for 1 h. The cells were washed with PBS twice again. 4′, 6-diamidino-2-phenylindole (DAPI) (Roche Company, Germany) with the proportion of 1:1000 was used to dilute and dye the cells. Then the cells were incubated at room temperature away from light for 10 min. The cells were washed with PBS (twice) again. Confocal microscope (Olympus Corporation of Japan, Model Number FV1200) was used to observe and take photos.

### Cell transfection

The SGC-7901 and KATO-III cells were divided into several groups: the blank group (without transfection sequence), negative control (NC) group (transfected with negative control sequence), miR-21 inhibitor group (transfected with miR-21 inhibitors), PTEN-siRNA group (transfected with PTEN siRNA) and miR-21 inhibitors + siRNA group (transfected both miR-21 inhibitors and PTEN siRNA). Cells were seeded in 25 cm^2^ culture flask and grew in complete medium to the density of 30 to 50%. Lipofectamin 2000 5 μl (Invitrogen Company, USA) was diluted by 100 μl serum-free medium and then was put at room temperature for 5 min. DNA1 μg was diluted by 100 μl serum-free culture medium. The two dilutions were mixed gently and rested at room temperature for 20 min for complex formation (combination of DNA and liposome) and serum-free culture medium was used to wash cells. Serum-free culture medium (without antibiotics) was added into the complex and then the complex was transferred into culture flask for transfection at 37°C, in 5% CO_2_. Complete medium was added 6∼8 h later and the cells were cultivated continuously.

### Western blotting

The SGC-7901 and KATO-III cells (5 × 10^5^ cells/well) were seeded in a 6-well culture plate. After cells being induced by TGF-β1 for 48 h, the cell incubation was stopped. Then 1 × sodium dodecyl sulfate (SDS) lysis was added into the cells and the protein extracts were heated at 100°C for 5 min for extraction of load sample. Polyacrylamide gel electrophoresis 10% was performed and transferred to polyvinylidenedifluoride (PVDF) membrane; voltage was 48V and the duration was 3.5 h. The cells were shaken and sealed by BSA5% at room temperature for 2 h and then washed by 1 × tris-buffered saline tween (TBST). BSA5% combining with E-cadherin, N-cadherin, β-catenin, Vimentin, Slug, PTEN, Akt, p-Akt and β-actin (CST Company, USA) was added and the cells were shaken and incubated at room temperature for 1 h and then washed by 1 × TBST. The secondary antibodies of goat anti-mouse and goat anti-rabbit (Abcam Company, UK) were added in to the cells, which were shaken and incubated at room temperature for 1 h and then washed by 1 × TBST. Electrogenerated chemiluminescence (ECL) developer solution was used to develop. Relative optical density of all immunoblot bands was analyzed. As mentioned above, Gene expressions of EMT related factors and PTEN were also detected by the qRT-PCR assay.

### Scratch test

After digesting into a single cell suspension, transfected cells were inoculated into a 6-well plate at a concentration of 10^6^ cells/well overnight, and scratched vertically with a 100 ul micro pipette tip on the next day. Thereafter, cells were washed twice with PBS and placed in serum-free culture medium. After 24 h and 48 h, cells were counted under an invert phase-contrast microscope in five random fields. Each migration test was run in triplicate.

### Xenograft tumor experiment in nude mice

A total of 36 4-week-old BALB/c nude mice were provided by Shanghai Laboratory Animal Center, Chinese Academy of Sciences (Shanghai, China). GC cells in logarithmic growth phase were digested using 0.25% trypsin, washed twice with PBS, followed by supernatant removal. The prepared single cell suspension was injected into subcutaneous right hip at a concentration of 0.2 ml/mouse to establish a xenograft tumor nude mice model. The 36 nude mice were divided into three groups with 6 mice in each group: the blank group, NC group, and miR-21 inhibitors group. The growth curve of xenograft tumors was drawn. The longest diameter (L) and the shortest diameter (W) were measured with a vernier caliper to calculate tumor volume (V) every day, and the growth curve was drawn again after treatment. After 28 d, tumors were separated completely, photographed and weighted. Fixed with formaldehyde, tumors were embedded with paraffin and sliced. Immunohistochemistry was used to detect the expressions of E-cadherin, N-cadherin, β-catenin, Vimentin, Slug and PTEN proteins.

### Statistical methods

SPSS 18.0 (SPSS Inc., Chicago, IL, USA) statistical software was used to analyze data. Measurement data were expressed as mean value ± standard deviation (x ± s). The comparison between groups of measurement data was analyzed by LSD-*t* test and the comparison among groups was analyzed by analysis of variance (ANOVA) analysis. Quantitation data were presented as frequency or rate. The comparison of categorical data was analyzed by chi-square test and the comparison of grading data using rank sum test. A *P* values less than 0.05 was considered as statistically significant.
